The article "Acyclovir Combined with Naloxone in the Treatment of Viral Encephalitis: A Meta-Analysis" was retracted in 2023. Reasons: unreliable results or conclusions; concerns about the data; concerns about the peer review; concerns about the citations.

# Acyclovir Combined with Naloxone in the Treatment of Viral Encephalitis: A Meta-Analysis

**DOI:** 10.1155/2022/8593251

**Published:** 2022-04-01

**Authors:** Wei Wang, Qing Zhao, Qifan Zhang

**Affiliations:** Department of Neurology, People's Hospital of Ningxia Hui Autonomous Region, Yinchuang, Ningxia Hui Autonomous Region 750002, China

## Abstract

**Background:**

The aim of this study was to systematically evaluate the efficacy and prognosis of acyclovir combined with naloxone in the treatment of patients with viral encephalitis (VE).

**Methods:**

PubMed, Web of Science, Embase, CNKI, and WanFang Data were searched for relevant literature published between 2000 and 2021. Meta-analysis was performed using Stata16.0 software. The treatment group was treated with acyclovir combined with naloxone, and the control group was treated with acyclovir alone.

**Results:**

A total of 12 studies with 986 participants were included. Compared with the control group, the treatment group could not only significantly improve the treatment response rate (OR = 5.53, 95% CI: 3.50, 8.74; *P* ≤ 0.001), but also reduce the incidence of adverse reactions (OR = 0.25, 95% CI: 0.17, 0.38; *P* ≤ 0.001). In addition, the combined treatment significantly inhibited the levels of inflammatory factors and neuron-specific enolase (NSE) in VE patients. The time for cerebrospinal fluid to return to normal (SMD = −2.73, 95% CI: −2.96, −2.51; *P* ≤ 0.001), as well as the disappearance time of meningeal irritation (SMD = −3.58, 95% CI: −4.96, −2.20; *P* ≤ 0.001), headache (SMD = −3.87, 95% CI: −5.84, −1.91; *P* ≤ 0.001), convulsion (SMD = −3.65, 95% CI: −4.56, −2.75; *P* < 0.001), tic (SMD = −4.083, 95% CI: −5.18, −2.98; *P* ≤ 0.001) and disturbance of consciousness (SMD = −4.96, 95% CI: −6.28, −3.63; *P* ≤ 0.001) in the treatment group were significantly shorter than those in the control group.

**Conclusion:**

A combination of acyclovir and naloxone can reduce the inflammatory response and shorter the time to symptom relief and disappearance, which is worthy of clinical promotion.

## 1. Introduction

Viral encephalitis (VE) is a life-threatening consequence of central nervous system infections caused by viruses, with high morbidity, mortality and disability [1]. In China, human enteroviruses are the main pathogens of VE, followed by herpes simplex virus (HSV), Japanese encephalitis virus (JEV) [2, 3]. Its common clinical features are fever, headache, nausea, vomiting, meningeal irritation signs and cerebrospinal fluid changes; in severe cases, VE leads to loss of consciousness, seizures and focal neurological deficits, and pleocytosis of cerebrospinal fluid [4–6]. According to the survey, the mortality rate of VE in China is 3.13% [7]. In developing countries, about 50–60% of VE patients have a poor prognosis [8, 9], such as neurological deficits as well as cognitive, affective, and behavioral dysfunction, placing great economic and mental stress on patients' families and society [10]. Therefore, it is particularly vital to find effective methods for early diagnosis and treatment of VE and consequently to improve prognosis.

The article "Acyclovir Combined with Naloxone in the Treatment of Viral Encephalitis: A Meta-Analysis" was retracted in 2023. Reasons: unreliable results or conclusions; concerns about the data; concerns about the peer review; concerns about the citations.

The primary clinical treatment measures for VE include supportive treatment and antiviral therapy [11]. The latter is achieved through antiviral drugs, such as acyclovir, prednisolone, and ganciclovir [12]. Acyclovir is a classic drug for empirical treatment of VE, which is a nucleotide analogue with antiviral activity against HSV and related viruses [13]. If the possibility of VE cannot be ruled out 6 hours after admission, it is recommended to start initial treatment with acyclovir. However, acyclovir alone has a limited antiviral range, and long-term use of acyclovir is prone to drug resistance [14]. Additionally, up to 20% of patients treated with acyclovir develop nephropathy and adverse reactions [15]. Naloxone is an opioid receptor antagonist, and is an effective drug for VE [16]. However, long-term and high-dose administration of naloxone may cause arrhythmia, cardiogenic pulmonary edema and even myocardial infarction [17]. Many scholars believe that clinically, a combination of acyclovir and naloxone can effectively relieve the inflammatory response and brain injury caused by VE, and can protect neuronal cells; the combination has a small risk of sequelae, and is conducive to the outcome of the disease [18]. Liu et al. [19] also confirmed that naloxone combined with acyclovir was more effective than each drug alone in the treatment of VE in children, with lower incidence rates of adverse reactions and sequelae. Although relevant studies have been conducted to analyze and compare the effects of the two drug combinations, they are often limited by the number of patients and do not provide enough evidence to confirm the safety and efficacy of acyclovir and naloxone combination therapy. As a result, the current study was conducted on evidence-based medicine and a review of national and worldwide evidence on VE drug therapy. By analyzing indicators such as treatment response rate, the incidence of adverse effects, inflammatory factor levels, symptom relief and time to symptom relief and disappearance, the collected data were summarized and evaluated using meta-analysis to provide more sufficient evidence and new strategies for the rational use of drugs for VE.

## 2. Methods

### 2.1. Literature Retrieval

PubMed, Web of Science, Embase, China National Knowledge Infrastructure, and WanFang Data were searched for relevant articles published between 2000 and 2021. The search terms were set as: “viral encephalitis”, “acyclovir”, and “naloxone”.

The article "Acyclovir Combined with Naloxone in the Treatment of Viral Encephalitis: A Meta-Analysis" was retracted in 2023. Reasons: unreliable results or conclusions; concerns about the data; concerns about the peer review; concerns about the citations.

### 2.2. Exclusion Criteria

The followings were excluded: (1) review, conference paper, abstract, case report; (2) before-after study in the same patients; (3) literature lacking basic data; (4) literature without a control group; (5) duplicate literature, systematic review and animal experiment.

### 2.3. Inclusion Criteria

Literature that met the following criteria were included: (1) Study subjects: Patients clinically diagnosed with VE, and met the diagnostic criteria for VE [7], without gender or nationality restrictions. (2) Interventions: The control group was treated with acyclovir, and the treatment group was treated with acyclovir combined with naloxone. (3) Outcome measures: treatment response rate, the incidence of adverse reactions; levels of tumor necrosis factor-*α* (TNF-*α*), interleukin-1 (IL-1), interleukin-6 (IL-6) and neuron-specific enolase (NSE) after treatment; time for cerebrospinal fluid to return to normal, disappearance time of meningeal irritation, disappearance time of headache, disappearance time of convulsion, disappearance time of tic, disappearance time of disturbance of consciousness after treatment.

### 2.4. Data Extraction

Two researchers independently reviewed the retrieved articles and collected the data including the name of the first author, year of publication, basic information of the subjects (age, gender, etc.), study design, main results. All articles were jointly decided for inclusion or not by the two researchers, and disagreements were resolved by discussion with a third party.

### 2.5. Statistical Analysis

Statistical analysis of all data was performed using Stata16.0 software. Standard mean difference (SMD) was as an effect size for continuous data, while odds ratio (OR) and 95% confidence interval (CI) for categorical variables. The heterogeneity of included studies was assessed using Cochrane's *Q* test and I^2^ statistics. When *P* > 0.1 or I^2^ < 50%, a fixed-effect model was used for meta-analysis, otherwise a random-effect model was adopted for analysis (*P* > 0.10 or I^2^ < 50%). Funnel plot and Begg's test were used to evaluate the publication bias of the studies, and sensitivity analyses to assess the stability of the results.

## 3. Results

### 3.1. Result of Literature Retrieval

The literature screening process is shown in Figure 1. A total of 424 articles were initially retrieved, and then 351 duplicated articles were removed. Subsequently, 41 articles were excluded by titles or abstracts. After further reading the full text, 20 literature with insufficient data or duplicated data were excluded. Finally, 12 articles were included [18–29] for meta-analysis. The included studies were randomized controlled clinical studies, including 986 study subjects, 496 in the treatment group and 490 in the control group. The basic characteristics of the included literature are shown in Table 1.

The article "Acyclovir Combined with Naloxone in the Treatment of Viral Encephalitis: A Meta-Analysis" was retracted in 2023. Reasons: unreliable results or conclusions; concerns about the data; concerns about the peer review; concerns about the citations.

### 3.2. Comparison of Response Rate and Incidence of Adverse Reactions after Treatment

Eleven included studies compared the response rate between the two groups [19–29]. No marked heterogeneity was found among the included studies (*P* = 0.999, I^2^ = 0.0%), so a fixed-effect model was used for meta-analysis. Nine included studies compared the incidence rate of adverse reactions between the two groups [18–23, 25, 27, 28]. No significant heterogeneity was identified among the included studies (*P* = 0.704, I^2^ = 0.0%), so a fixed-effect model was employed for analysis. The results showed in comparison with the control group, the combination treatment significantly increased the effective rate (OR = 5.53, 95% CI: 3.50, 8.74; *P* ≤ 0.001, Figure 2(a)), and markedly decreased the incidence rate of adverse reactions (OR = 0.25, 95% CI: 0.17, 0.38; *P* ≤ 0.001, Figure 2(b)).

Funnel plot and Begg's test were further adopted for confirming whether publication bias existed in the included studies. According to the funnel plots, the studies regarding response rate (Figure 3(a)) and the incidence of adverse reactions (Figure 3(b)) showed a symmetrical distribution, respectively; *P* values of the Begg test were 0.507 and 0.404, respectively. The above indicated no publication bias in the included studies.

Sensitivity analysis by excluding each study one by one revealed that the pooled effect sizes of the treatment response rate (Figure 4(a)) and the incidence of adverse reactions (Figure 4(b)) fluctuated within (3.31, 8.74) and (0.17, 0.38), respectively, indicating low sensitivity and confirming that the results of this meta-analysis were robust and credible.

### 3.3. Comparison of Inflammatory Factors and Neuron-specific Enolase (NSE) Levels after Treatment

The changes of inflammatory factors and NSE levels after treatment were analyzed. Significant heterogeneity was identified among the included studies regarding TNF-*α* (*P* < 0.05; I^2^ = 96.1%), IL-1 (*P* < 0.05; I^2^ = 72.2%), IL-6 (*P* < 0.05; I^2^ = 76.7%), and NSE (*P* < 0.05; I^2^ = 95.0%), respectively, so each indicator was analyzed using a random-effect model.

Seven studies [18, 23, 24, 26–29] compared TNF-*α* levels after treatment between the two groups. In comparison with the control group, a combination of acyclovir and naloxone could achieve a significantly lower TNF-*α* level after treatment (SMD = −3.64, 95% CI: −4.89, −2.38; *P* ≤ 0.001; Figure 5(a)).

The article "Acyclovir Combined with Naloxone in the Treatment of Viral Encephalitis: A Meta-Analysis" was retracted in 2023. Reasons: unreliable results or conclusions; concerns about the data; concerns about the peer review; concerns about the citations.

Seven studies [18, 19, 23, 26–29] compared IL-1 levels after treatment between the two groups. The results showed that the IL-1 level in the treatment group was significantly lower than that in the control group (SMD = −1.62, 95% CI: −1.98, −1.25; *P* ≤ 0.001; Figure 5(b)).

Four articles [18, 19, 26, 28] compared IL-6 levels after treatment between the two groups. A marked reduction of IL-6 level was found the treatment group compared with the control group (SMD = −1.54, 95% CI: −2.08, −1.01; *P* < 0.001; Figure 5(c)).

Five studies [18, 20–22, 24] compared NSE levels after treatment between the two groups. Compared with the control group, the NSE level in the treatment group was decreased (SMD = −2.51, 95% CI: −3.58, −1.44; *P* ≤ 0.001; Figure 5(d)).

Sensitivity analysis by excluding each study one by one revealed that the range of pooled effect sizes of TNF-*α* (Figure 6(a)), IL-1 (Figure 6(b)), IL-6 (Figure 6(c)), and NSE (Figure 6(d)) did not change much, respectively. Although the results of TNF-*α* by Jiang et al. and NSE results by Dong et al. exceeded the original CIs, no opposite results occurred. The above suggested low sensitivity and confirmed the results of this meta-analysis were robust and credible.

### 3.4. Comparison of Time to Symptom Relief after Treatment

Seven studies [20, 22, 23, 25–28] reported the time for cerebrospinal fluid to return to normal after treatment. By using a fixed-effect model (*P* = 0.061; I^2^ = 50.1%) for pooling the effect size, the result showed that in comparison with the control group, a combination of acyclovir and naloxone contributed to significantly shorten the time for cerebrospinal fluid to return to normal (SMD = −2.73, 95% CI: −2.96, −2.51; *P* ≤ 0.001; Figure 7(a)).

Five articles [20, 23, 24, 26, 28] compared the disappearance time of meningeal irritation after treatment. By using a random-effects model (*P* < 0.05; I^2^ = 95.0%), the result revealed that after treatment, meningeal irritation in the treatment group disappeared markedly earlier than that in the control group (SMD = −3.58, 95% CI: −4.96, −2.20; *P* ≤ 0.001; Figure 7(b)).

Sensitivity analysis revealed that pooled effect sizes of time for cerebrospinal fluid to return to normal (Figure 8(a)) and disappearance time of meningeal irritation (Figure 8(b)) did not change much by excluding each study one by one, indicating low sensitivity and confirming that the results of this meta-analysis were robust and credible.

### 3.5. Comparison of Symptom Disappearance Time after Treatment

Significant heterogeneity was identified among the included studies regarding disappearance time of headache (*P* < 0.05; I^2^ = 98.5%), disappearance time of convulsion (*P* < 0.05; I^2^ = 92.6%), disappearance time of tic (*P* < 0.05; I^2^ = 95.4%) and disappearance time of disturbance of consciousness (*P* < 0.05; I^2^ = 96.2%) after treatment, so each indicator was analyzed using a random-effect model.

The article "Acyclovir Combined with Naloxone in the Treatment of Viral Encephalitis: A Meta-Analysis" was retracted in 2023. Reasons: unreliable results or conclusions; concerns about the data; concerns about the peer review; concerns about the citations.

Nine studies [20–28] compared disappearance time of headache, tic and disturbance of consciousness after treatment. Eight studies [20, 22–28] compared disappearance time of convulsion after treatment. Meta-analysis results showed that after treatment, headache (SMD = −3.87, 95% CI: −5.84, −1.91; *P* ≤ 0.001; Figure 9(a)), convulsion (SMD = −3.65, 95% CI: −4.56, −2.75; *P* < 0.001; Figure 9(b)), tic (SMD = −4.08, 95% CI: −5.18, −2.98; *P* ≤ 0.001; Figure 9(c)), and disturbance of consciousness (SMD = −4.96, 95% CI: −6.28, −3.63; *P* ≤ 0.001; Figure 9(d)) in the patients of the treatment group disappeared significantly earlier that those in the control group.

Sensitivity analysis revealed (Figures 10(a)–10(d)) that pooled effect sizes did not change much after excluding each study one by one, indicating low sensitivity and confirming that the results of this meta-analysis were robust and credible.

## 4. Discussion

VE is a central nervous system disease caused by common infectious viruses and HSV [7], with high incidence, complex condition, rapid progression and poor prognosis [6]. With the progress of science and technology, the current medical treatment can effectively control the condition, but there has been controversy in the use of drugs. Some scholars believe that virus-caused diseases need to effectively kill the viruses to achieve therapeutic effects [6, 8]. Therefore, acyclovir has become the optimal choice for clinical medication. However, acyclovir alone can only kill HSV [30], but is ineffective against other common infectious viruses [31]. Additionally, acyclovir can cause symptomatic bradycardia and other common side effects, such as nausea, diarrhea, headache, dizziness, and mental changes [32, 33]. Naloxone is a pure narcotic antagonist, which is a relatively safe and effective drug for treating brain diseases, and for reversing anesthesia-related cardiovascular and respiratory depression [34]. But naloxone may sometimes bring about non-narcotic overdose [34], and causes adverse effects including hypertension, ventricular arrhythmias, sudden cardiac arrest, seizures, and rarely pulmonary edema [35]. A combination of acyclovir and naloxone not only exerts the effectiveness of both drugs, but may also compensate for the limitations of naloxone in clinical practice [19]. In this study, by using meta-analysis, we analyzed randomized controlled studies on acyclovir alone and its combination with naloxone in the treatment of viral encephalitis. A total of 12 studies with 986 participants were included. Eleven of the included studies compared response rates between the two groups, and nine of the included studies compared the incidence of adverse reactions between the two groups. No significant heterogeneity was found in the included studies. The results showed that the combination treatment significantly increased the efficiency and significantly decreased the incidence of adverse reactions compared to the control group. Further analysis showed no publication bias in the included studies. Sensitivity analysis performed by excluding each study individually showed that the combined effect sizes for treatment response rate and incidence of adverse effects fluctuated within the ranges of (3.31, 8.74) and (0.17, 0.38), respectively, indicating low sensitivity and reconfirming the robustness and reliability of the results of the meta-analysis.

The article "Acyclovir Combined with Naloxone in the Treatment of Viral Encephalitis: A Meta-Analysis" was retracted in 2023. Reasons: unreliable results or conclusions; concerns about the data; concerns about the peer review; concerns about the citations.

VE can trigger, mediate, or participate in the inflammatory response, which promotes the production and release of inflammation-related factors (e.g., TNF-*α*, IL-1, IL-6) [19]. Studies have shown that the production of TNF-*α* in the brain promotes the progression of neurotoxicity and encephalitis [36]. IL-1 has been proved to play a crucial role in the pathogenesis of inflammation in most autoinflammatory diseases [37]. IL-6 is a pleiotropic cytokine with a wide range of roles in integrated immune responses, and it has different effects on immune activity through classical or trans-signaling pathways [38]. NSE level is currently one of the clinically recognized markers reflecting neuronal damage [39, 40]. In this study, we found that the levels of TNF-*α*, IL-1, IL-6 and NSE in VE patients treated with the combined therapy were significantly lower than those in patients treated with acyclovir alone. It is suggested that combined treatment resulted in a significant improvement in the inflammatory response, and has a good anti-inflammatory effect [26].

This study also found that compared to the control group, combined treatment can significantly shorten the time of clinical symptom relief and the time of disappearance of adverse reactions. Specifically, a combination of acyclovir and naloxone significantly shortens the disappearance time of headache, convulsion, tic and disturbance of consciousness. This indicates that the combined treatment can promote the rapid relief and disappearance of various symptoms of VE and yet again, appears to have superior clinical outcomes.

The article "Acyclovir Combined with Naloxone in the Treatment of Viral Encephalitis: A Meta-Analysis" was retracted in 2023. Reasons: unreliable results or conclusions; concerns about the data; concerns about the peer review; concerns about the citations.

Compared with previous studies, the advantages of this study include two aspects. First, more specific comprehensive indicators of clinical efficacy and prognosis. This study obtains more comprehensive and persuasive results by analyzing the indicators including treatment response rate, incidence of adverse reactions, inflammatory factor levels, symptom relief and time to symptom relief and disappearance. Second, only randomized controlled trials. This kind of trial has a clear causal relationship between a treatment and an outcome, and can effectively avoid the effect of potential unknown factors on the trial results.

Viral encephalitis is difficult to treat [6–8]. In the 1980s, the advent of acyclovir therapy changed the outcome of HSV encephalitis [3]. However, patients are still dying as a result of the disease, and many survivors are left with devastating side effects [6–9]. For some years evidence from *in vitro* and animal models has shown that adding corticosteroids to acyclovir for the treatment of VE may enhance outcomes [12–14]. Attempts have been made to use immunoglobulin therapy with limited effects. Randomized controlled studies are needed to determine if intravenous immunoglobulin is beneficial as a first-line treatment [41]. Immune responses in encephalitis may be clarified using novel laboratory approaches such as proteomics, transcriptomics, and metabolomics, which might assist to stratify unknown patients into aetiological groups [41, 42]. In addition, the use of next-generation sequencing to search for putative infectious agents and the use of protein arrays and mass spectrometry to search for novel antibodies may provide a basis for diagnosis and treatment for more patients in the future [42]. As a result, new therapeutic procedures are desperately needed to increase treatment response rates and limit the occurrence of adverse effects. Our findings indicate that combination treatment has higher therapeutic efficacy and a lower risk of side effects. It contributed to the existing of data supporting the use of acyclovir in combination with naloxone in the treatment of VE and broadens the idea of further improving the current status of VE treatment.

## 5. Conclusion

Compared with acyclovir alone, acyclovir combined with naloxone is more effective in the treatment of VE, with lower adverse reactions. Additionally, the latter can reduce inflammatory response and shorter the time to symptom relief and disappearance. Therefore, this combined treatment is worthy of being widely popularized in clinical application.

## Figures and Tables

**Figure 1:** Flow diagram of literature screening.

The article "Acyclovir Combined with Naloxone in the Treatment of Viral Encephalitis: A Meta-Analysis" was retracted in 2023. Reasons: unreliable results or conclusions; concerns about the data; concerns about the peer review; concerns about the citations.

**Figure 2:** Forest plots of treatment response rate (a) and incidence of adverse reactions (b) after treatment for viral encephalitis.

**Figure 3:** Funnel plots of treatment response rate (a) and incidence of adverse reactions (b) after treatment for viral encephalitis.

**Figure 4:** Sensitivity analysis of treatment response rate (a) and incidence of adverse reactions (b) after treatment for viral encephalitis.

**Figure 5:** Forest plots of TNF-*α* (a), IL-1 (b), IL-6 (c), and NSE (d) levels in the two groups after treatment for viral encephalitis.

**Figure 6:** Sensitivity analysis of TNF-*α* (a), IL-1 (b), IL-6 (c), and NSE (d) levels in the two groups after treatment for viral encephalitis.

**Figure 7:** Forest plots of time for cerebrospinal fluid to return to normal (a) and disappearance time of meningeal irritation (b) after drug treatment for viral encephalitis.

**Figure 8:** Sensitivity analysis of time for cerebrospinal fluid to return to normal (a) and disappearance time of meningeal irritation (b) after drug treatment for viral encephalitis.

**Figure 9:** Forest plots of symptom disappearance time after drug treatment for viral encephalitis (a) headache disappearance time, (b) convulsion disappearance time, (c) tic disappearance time, (d) disturbance of consciousness disappearance time.

**Figure 10:** Sensitivity analysis of symptom disappearance time after drug treatment for viral encephalitis (a) headache disappearance time, (b) convulsion disappearance time, (c) tic disappearance time, (d) disturbance of consciousness disappearance time.

**Table 1:** Basic characteristics of included literature.

Study	Year	Sample time (year month)	Cases treat/Con	Age (years)		Disease (days)		Sex (male/female)		Study design	Outcome measures
				Treat group	Con group	Treat group	Con group	Treat group	Con group		
Shi chunxiang	2021	2017.01–2018.03	45/45	7.2 ± 2.5	7.1 ± 2.3	3.5 ± 0.4	3.5 ± 0.4	26/19	24/21	RCT	②③④⑥
Li huiying	2014	2010.06–2012.06	62/62	6.7 ± 2.4	7.3 ± 3.2	3.2 ± 0.4	3.7 ± 0.6	34/28	32/32	RCT	①②⑥⑦⑧⑨⑩⑪⑫
Dong xuezheng	2017	2015.01–2016.12	29/29	31.1 ± 2.7	32.4 ± 2.3	NP	NP	16/13	17/12	RCT	①②⑥⑨⑪⑫
Ding hongliang	2018	2016.03–2017.03	49/49	5.8 ± 3.3	5.7 ± 3.2	2.6 ± 1.2	2.4 ± 1.1	30/19	28/21	RCT	①②⑥⑦⑨⑩⑪⑫
Li xinsheng	2018	2016.08–2017.08	36/36	5.3 ± 1.7	5.4 ± 1.7	NP	NP	19/17	20/16	RCT	①②③④⑤⑦⑧⑨⑩⑪⑫
Jiang zonghua	2019	2015.07–2018.07	43/43	5.3 ± 1.5	5.1 ± 1.5	2.1 ± 0.6	2.0 ± 0.5	25/18	24/19	RCT	①③⑥⑧⑨⑩⑪⑫
Xiao yuehong	2016	2015.01–2016.09	30/30	6.8 ± 2.3	6.9 ± 2.8	3.2 ± 0.4	3.3 ± 0.4	18/12	15/15	RCT	①②⑦⑨⑩⑪⑫
Wu ting	2018	2016.07–2017.06	30/30	5.2 ± 1.5	5.3 ± 1.4	2.2 ± 0.4	2.1 ± 0.3	17/13	18/12	RCT	①③④⑤⑦⑧⑨⑩⑪⑫
Sun weiwei	2013	2010.03–2013.02	44/44	4.9 ± 2.7	5.0 ± 2.5	2.2 ± 0.5	2.3 ± 0.4	26/18	25/19	RCT	①②③④⑦⑨⑩⑪⑫
Ruan tao	2016	2013.05–2014.08	40/40	5.2 ± 2.5	5.3 ± 2.6	NP	NP	23/17	22/18	RCT	①②③④⑤⑦⑧⑨⑩⑪⑫
Zeng yuan	2019	2017.02–2018.05	37/37	5.4 ± 3.3	5.2 ± 3.3	2.7 ± 1.4	2.5 ± 1.2	18/19	19/18	RCT	①③④
L. NIU	2020	2013.07–2014.01	51/45	2.9 ± 2.6	2.8 ± 2.5	3.3 ± 0.6	3.3 ± 0.5	33/18	28/17	RCT	①②④⑤

Note. Treat: Treatment; Con : Control; RCT: randomized controlled trial; NR : Not reported; ①: Effective rate; ②: Adverse effects rate; ③: Tumor necrosis factor-*α* level after treatment; ④: Interleukin-1 level after treatment; ⑤: Interleukin-6 level after treatment; ⑥: Neuron enolase level after treatment; ⑦: Time for cerebrospinal fluid to return to normal after treatment; ⑧: Disappearance time of meningeal irritation after treatment; ⑨: Disappearance time of headache after treatment; ⑩: Disappearance time of convulsion after treatment; ⑪: disappearance time of tic after treatment; ⑫: Disappearance time of disturbance of consciousness after treatment.

The article "Acyclovir Combined with Naloxone in the Treatment of Viral Encephalitis: A Meta-Analysis" was retracted in 2023. Reasons: unreliable results or conclusions; concerns about the data; concerns about the peer review; concerns about the citations.

## Data Availability

The data used to support the findings of this study are available from the corresponding author upon request.
